# Isoflavaspidic Acid PB Extracted from *Dryopteris fragrans* (L.) Schott Inhibits *Trichophyton rubrum* Growth via Membrane Permeability Alternation and Ergosterol Biosynthesis Disruption

**DOI:** 10.1155/2022/6230193

**Published:** 2022-06-24

**Authors:** Zhisi Zhang, Xueping Liu, Zhibin Shen, Yanfen Chen, Cong Chen, Ying SiTu, Chunping Tang, Tao Jiang

**Affiliations:** ^1^School of Traditional Chinese Medicine, Guangdong Pharmaceutical University, Guangzhou, 510006 Guangdong, China; ^2^Guangdong Provincial Engineering Center of Topical Precise Drug Delivery System, Guangdong Pharmaceutical University, Guangzhou, 510006 Guangdong, China; ^3^Laboratory Animal Center, Guangdong Pharmaceutical University, Guangzhou, 510006 Guangdong, China; ^4^Guangzhou Key Laboratory of Construction and Application of New Drug Screening Model Systems, Guangzhou 510006, China

## Abstract

Isoflavaspidic acid PB (PB), a phloroglucinol derivative extracted from aerial parts of *Dryopteris fragrans* (L.) Schott, had antifungal activity against several dermatophytes. This study was aimed at exploring the antifungal mechanism of PB against *Trichophyton rubrum* (*T. rubrum*). The effectiveness of PB in inhibiting *T. rubrum* growth was detected by time-kill kinetics study and fungal biomass determination. Studies on the mechanism of action were investigated using scanning electron microscopy (SEM), transmission electron microscopy (TEM), sorbitol and ergosterol assay, nucleotide leakage measurement, and UPLC-based test and enzyme-linked immunosorbent assay. Fungicidal activity of PB was concentration- and time-dependent at 2 × MIC (MIC: 20 *μ*g/mL) after 36 h. The total biomass of *T. rubrum* was reduced by 64.17%, 77.65%, and 84.71% in the presence of PB at 0.5 × MIC, 1 × MIC, and 2 × MIC, respectively. SEM analysis showed that PB changed mycelial morphology, such as shrinking, twisting, collapsing, and even flattening. TEM images of treated cells exhibited abnormal distributions of polysaccharide particles, plasmolysis, and cytoplasmic content degradation accompanied by plasmalemma disruption. There were no changes in the MIC of PB in the presence of sorbitol. However, the MIC values of PB were increased by 4-fold with exogenous ergosterol. At 4 h and 8 h, PB increased nucleotide leakage. Besides, ergosterol content in *T. rubrum* membrane treated with PB at 0.5 × MIC, 1 × MIC, and 2 × MIC was decreased by 9.58%, 15.31%, and 76.24%, respectively. There was a dose-dependent decrease in the squalene epoxidase (SE) activity. And the reduction in the sterol 14*α*-demethylase P450 (CYP51) activity was achieved after PB treatments at 1 × MIC and 2 × MIC. These results suggest that PB displays nonspecific action on the cell wall. The membrane damaging effects of PB were attributed to binding with ergosterol to increase membrane permeability and interfering ergosterol biosynthesis involved with the reduction of SE and CYP51 activities. Further study is needed to develop PB as a natural antifungal candidate for clinical use.

## 1. Introduction

Superficial mycoses have affected about 20-25% of the worldwide population with incidence, in particular those involving dermatophyte infection, having increased in the recent decades [1, 2]. Dermatophytosis are infections of the stratum corneum or keratinized adnexal structures caused by dermatophytes [3]. Typical lesions of the infected skin are clinically manifested as scaly, alopecia, swelling, and even deep tissue infection such as granulomas in severe cases [4]. As the special fungi in keratin degradation, dermatophytes belong to three genera: *Trichophyton*, *Epidermophyton*, and *Microsporum* [5]. *Trichophyton rubrum* is the main etiological agent, accounting for about 70% of dermatophytosis [6].

Currently, controlling dermatophytosis primarily relies on several classes of commercial antidermatophytic drugs, including polyenes (amphotericin B), azoles (miconazole, ketoconazole, and fluconazole), allylamines (terbinafine), and echinocandins (caspofungin, anidulafungin) [7]. Despite progress in antidermatophytic therapy, prolonged duration of treatment, resistance problems, and a narrow spectrum of activity severely limit the effectiveness of available antifungals [8, 9]. Unfortunately, some are fungistatic rather than fungicidal [10]. Moreover, many of them have a certain toxicity to patients, such as hepatotoxicity of azoles, cardiopathy of echinocandins, and nephrotoxicity of amphotericin B [11]. In this context, there is an urgent demand for new antifungal agents that are more effective against target dermatophytes and less toxic for host cells.

*Dryopteris fragrans* (L.) Schott (*D. fragrans*), a deciduous perennial herb, belongs to family Dryopteridaceae and broadly distributes in Asia-temperate, Europe and North America [12, 13]. Infusions and decoctions of its aerial parts are folk medicines that have been used in a wide range of curing fungal skin infections, such as dermatitis, rashes, psoriasis, and beriberi [14]. In order to remove dandruff and relieving itchiness, extraction solution has been applied for local residents in Wu-Da-Lian-Chi (Heilongjiang province, China) to wash hair [15].

Over the past few years, numerous scholars have focused on the screening of antifungal active ingredients from the aerial parts of *D. fragrans*. A series of phytochemical studies on this plant led to the identifications of phloroglucinols, terpenes, flavonoids, phenylpropanoids, etc. It has been reported that 95% ethanol extract was the most effective fraction of *D. fragrans*, which possessed fungistatic and fungicidal activities on *T. rubrum* [16]. Similarly, *Microsporum canis* (*M. canis*) was found to be sensitive to the effective fraction of *D. fragrans* both *in vivo* and *in vitro* [17, 18]. As discussed by Liu et al. [19], HPLC-ESI-MS analysis was undertaken to reveal that fourteen compounds belonging to phloroglucinol are the main active ingredients of the effective fraction of *D. fragrans*.

Isoflavaspidic acid PB (PB), a phloroglucinol derivative extracted from aerial parts of *D. fragrans*, had a broad spectrum of antifungal activity, with minimal inhibitory concentration values for a total of 25 dermatophyte strains between 20 and 40 *μ*g/mL [20, 21]. Our previous studies had also showed the antibiofilm activity of PB against dermatophytes by the inhibition of ergosterol biosynthesis [20]. The mechanisms of PB on biofilm biological activities were also associated with the inhibition of the biofilm adhesion and mRNA expression of ergosterol metabolism-related genes *ERG6* and *ERG11* [22]. However, the potential mechanism of PB against *T. rubrum* is still poorly explored. In this study, time–kill kinetics study, fungal biomass determination, scanning and transmission electron microscopy, sorbitol protection assay, ergosterol binding assay, intracellular leakage measurement, and ergosterol quantification assay, as well as the activities of squalene epoxidase and sterol 14*α*-demethylase, were performed to investigate the mode of action of PB against *T. rubrum* in vitro.

## 2. Materials and Methods

### 2.1. Fungal Strains and Culture Conditions

Two standard strains including *T. rubrum* (CMCC(F)T1d) and *Candida parapsilosis* (ATCC 22019) were obtained from the Institute of Dermatology, Chinese Academy of Medical Sciences, Nanjing, China. The strains were maintained at -70°C on Sabouraud Broth (Sigma Aldrich, St. Louis Missouri, USA) supplemented with 30% glycerol. Before conducting the experiments, these strains were reactivated and subcultured on the Sabouraud dextrose agar medium (SDA, OXOID Ltd, Basingstoke, Hampshire, UK) at 28°C until suitable conidiation. The SDA medium contained dextrose 20 g, agar 15 g, and peptone 10 g in 1.0 L of sterile water.

### 2.2. Inoculum Suspension Preparation

The inoculum suspension was prepared in accordance with the previous studies [23]. *T. rubrum* (CMCC(F)T1d) was grown on SDA at 28°C for 7 days. Fungal colonies were suspended in approximately 5 mL of phosphate buffer saline (PBS, 10 mM, pH 7.2) by gently rubbing them with the tip of a Pasteur pipette. The densities of these suspensions were adjusted to obtain the inoculum of 1 × 10^6^~5 × 10^6^ CFU/mL and confirmed by counting the microorganisms in a Neubauer chamber.

### 2.3. The Preparation of Relevant Antifungal Agents

Terbinafine (TBF, purity > 99%), amphotericin B (AMB, purity > 99%), and miconazole (MCZ, purity > 99%) were used as positive controls. They were obtained from Sigma-Aldrich Co. LLC. (Shanghai, China). The medicines were dissolved in dimethyl sulfoxide (DMSO, Baishi Chemical Industry Co. Ltd, Tianjin, China) to obtain an initial concentration of 6.4, 2, and 2 mg/mL, respectively, and kept at -20°C until use. The final concentration of DMSO did not exceed 0.5% in the assays, suggesting that it did not to interfere with fungal growth [24, 25].

### 2.4. Plant Material and Collection

Prof. De-Lian Zhang (D.-L.Z., Harbin University of Commerce, China) identified the *D. fragrans* sample taken in August 2017 in Wu-Da-Lian-Chi, Heilongjiang province, China (geographic coordinates, latitude: 48° 30′~48° 51′ N, longitude: 126° 00′~126° 25′ E). The plant's voucher specimen (registration number: XLMJ-201708) was deposited in the School of Traditional Chinese Medicine, Guangdong Pharmaceutical University.

### 2.5. Extraction and Isolation of PB

Ethanolic extract of aerial parts of *D. fragrans* and the subsequent PB isolation (purity > 95%) was carried out as previously described [21]. The air-dried aerial parts of *D. fragrans* were extracted by 50% ethanol three times under refluxing. The crude extract was preliminarily isolated by six gradients of silica gel column chromatography with a mobile phase of petroleum-acetone (100 : 1, 70 : 1, 50 : 1, 30 : 1, 10 : 1, and 1 : 1). Six fractions (Frs. A→F) were prepared in column chromatography. Frs. C were further applied to gel Sephadex LH-20 column (60-100 mesh), eluted with chloroform-methanol (1 : 1), and purified by preparative HPLC to obtain the final products. The molecular formula of PB was analyzed by ESI-MS analysis, and its chemical structure (Figure 1) was confirmed with the aid of different spectroscopic techniques (IR, ^1^H-NMR, and ^13^C-NMR).

### 2.6. Susceptibility Tests

Based on Clinical and Laboratory Standards Institute (CLSI) document (M38-A2), minimal inhibitory concentration (MIC) and minimal fungicidal concentration (MFC) values of PB against *T. rubrum* (CMCC(F)T1d) were investigated by broth microdilution method. For the MIC determination, the stock suspensions were diluted 1 : 100 in RPMI-1640 medium to obtain the final inoculum of 2 × 10^4^~5 × 10^4^ CFU/mL. Serial twofold dilutions were incorporated into these wells to yield final concentrations ranging from 0.6250 to 320 *μ*g/mL for PB and between 0.0625 and 32 *μ*g/mL for the AMB-treated group, 0.0039 and 2 *μ*g/mL for the TBF-treated group, and 0.0156 and 8 *μ*g/mL for the MCZ-treated group. Subsequently, 100 *μ*L of corresponding fungal suspensions were added to the 96-well microplates. Negative control (no medicines) was used in this study to verify conidia viability and susceptibility to DMSO (0.5%). Finally, the microplates were sealed aseptically and incubated at 35°C. A reading was made to evaluate MIC values after the appropriate incubation time. MIC was defined as the lowest drug concentration that was able to visually inhibit 100% fungal growth. *Candida parapsilosis* (ATCC 22019) was utilized as a quality control (QC) strain to confirm accuracy and duplicability of our tests (results were valid for MIC values of AMB ranging from 0.5 to 4.0 *μ*g/mL for QC strain).

For the MFC determination, aliquots of inoculum were taken away from the wells of no visible growth to petri dish containing SDA medium. The microplates were incubated at 28°C for 14 days. The MFC was defined as the lowest concentration resulting in no growth on subculture [26]. The assay was tested in triplicate.

### 2.7. Time-Kill Kinetics Study

To evaluate the dynamic fungicidal effect of PB on *T. rubrum*, time-kill kinetics was determined as previously described [27], with minor magnifications. The stock inoculum was adjusted to 2 × 10^4^~5 × 10^4^ CFU/mL in RPMI-1640 medium containing PB at 0.5 × MIC, 1 × MIC, and 2 × MIC along with positive control (TBF). Control growth without drugs was tested similarly. The suspensions were incubated at 30°C with continuous agitation (150 rpm). At different time intervals (0, 12, 24, 36, 48, 60, and 72 h), samples were removed from the tubes and diluted with RPMI-1640 medium. Then, aliquots of 10-fold dilution were spread uniformly onto the surface of SDA culture medium. After the appropriate time of incubation, colonies were analyzed through the plate colony counting technique. Time-kill curve took shape by plating log_10_ CFU/mL against time (h). Fungicidal activity was considered as reduction in growth more than 99.9% or >3log_10_ in CFU/mL from the initial inoculum [28].

### 2.8. Fungal Biomass Determination

For determining the effect of PB on mycelial growth, the total biomass of *T. rubrum* (CMCC(F)T1d) under different environments was assessed using a previous method [29], with slight modifications. Briefly, the inoculum of 2 × 10^4^~5 × 10^4^ CFU/mL was incubated with PB at the concentration of 0.5 × MIC, 1 × MIC, and 2 × MIC. Correspondingly, positive controls were made with TBF at the concentration of 1 × MIC. Drug-free RPMI-1640 medium with the strain was used as growth control. These resulting mixtures were incubated at 30°C for 7 days and transferred into previously weighted Eppendorf tubes. After centrifugation at 14000 × g for 20 min, pellet was collected and dried at 60°C for 3~6 h to reach a constant weight. The total biomass of mycelium was determined in triplicate using an analytic balance.

### 2.9. Scanning Electron Microscopy (SEM)

In order to identify the changes in the apparent structure of *T. rubrum* (CMCC(F)T1d), SEM observation was performed in accordance with previous research [30]. After exposure to PB (0.5 × MIC, 1 × MIC, and 2 × MIC) and TBF (1 × MIC), *T. rubrum* cells were fixed at 4°C with 2.5% (*v*/*v*) glutaraldehyde in PBS (0.01 M, pH 7.2) for 4 h. The fixed samples were washed with the same buffer twice each for 10 min and dehydrated through a graded ethanol series (50%, 70%, 80%, 90%, 95%, and 100%) for 15 min at room temperature. Finally, samples were subjected to critical point drying in liquid carbon dioxide (samdri-PVT-3D, Tousimis Research Corporation), coated with gold using ion sputtering device (Hitachi technology, Japan), and examined under a scanning electron microscope (Hitachi Technology, Japan).

### 2.10. Transmission Electron Microscopy (TEM)

Due to the changes observed in the internal structure of *T. rubrum* (CMCC(F)T1d), TEM observation was carried out as previously described [31]. In brief, the 7-day-old fungal inoculums on SDA medium containing PB (0.5 × MIC, 1 × MIC, and 2 × MIC) and TBF (1 × MIC) were prefixed in 2.5% glutaraldehyde in PBS (0.01 M, pH 7.2) at 4°C for 2~4 h. This is followed by washing three times in the same buffer, infiltrating 1% molten agar, and postfixing with 1% osmium tetroxide in PBS (0.01 M, pH 7.2) for 2 h at room temperature. After that, dehydration was achieved in a graded ethanol-acetone series (10% steps for 50%-90% ethanol each of 15 min, 100% ethanol three times for 15 min each, and acetone twice for 15 min each). The dehydrated specimens were embedded with Epon 812 and polymerized in Spurr's resin at 60°C for 48 h. Ultrathin sections (60~80 nm thick) were made by an ultramicrotome (Hitachi Technology, Japan), mounted on copper grids, and stained with uranyl acetate and lead citrate. These sections were finally investigated at an accelerating voltage of 80 KV using a transmission electron microscope (Hitachi Technology, Japan).

### 2.11. Sorbitol Protection Assay

To assess if the test product destroys the cell wall, sorbitol protection assay was performed using medium with and without sorbitol (control) as previously described [32]. The sorbitol (Sigma-Aldrich, Shanghai, China) was added to the culture medium in a final concentration of 0.8 M. MIC values of PB against *T. rubrum* (CMCC(F)T1d) were measured by using the broth microdilution method in 96-well microplates. The plates were incubated at 35°C, and the results of analysis made after 4 days. This assay was carried out in triplicate to calculate the geometric mean values.

### 2.12. Ergosterol Binding Assay

In order to determine whether the mechanism of PB was involved in binding to ergosterol in the fungal membrane, ergosterol binding assay was detected based on the previous method [33], with slight modification. The MIC of PB against *T. rubrum* (CMCC(F)T1d) was determined by broth microdilution techniques, in the absence and presence of ergosterol (Sigma-Aldrich, Shanghai, China) added to culture medium at a concentration of 400 *μ*g/mL. Since AMB has been known to affect ergosterol in the cytoplasmic membrane, it was used as a positive control. The plates were incubated at 35°C and counted after 4 days. Each result was expressed as geometric mean of triplicates.

### 2.13. Nucleotide Leakage Measurement

The leakage of nucleotides from *T. rubrum* (CMCC(F)T1d) was measured based on the method described previously [9, 34]. Fungal cells after 7-day growth on SDA medium, washed with 3-Morpholinopropanesulfoinc Acid buffer (MOPS, Sigma Chemical Co., Louis Missouri, USA) and resuspended in cold MOPS (pH 6.0), were used to prepare the inoculum at the density of 2 × 10^4^~5 × 10^4^ CFU/mL. Subsequently, aliquots of the fungal inoculum were exposed to PB (0.5 × MIC, 1 × MIC, and 2 × MIC) and TBF (1 × MIC), respectively. Growth control involved the equal amount of sterile distilled water replacing the drugs. Cultures were incubated at 35°C under agitation in an incubator shaker (H&Z Biologic Scientific Co., Ltd, Guangzhou, China). At different time intervals (4 h and 8 h), fungal cells were passed through 0.22 *μ*m filters and collected for absorbance analysis at 260 nm with a UV-visible spectrophotometer (SHIMADZU, Japan). Moreover, SDS (2%) was regarded as lysing agent, which produces 100% nucleotide leakage. Rate of nucleotide leakage was computed by comparing the test values with the lysing agent values. Results presented are the means of values from three independent assays.

### 2.14. Ergosterol Quantitation Assay

Ergosterol extraction and quantitation were performed by an UPLC-based test. This method was adapted from Lin et al. [20] in our group that has preliminarily investigated the effect of PB on ergosterol content of *T. rubrum* mature biofilm. Initially, fungal suspensions with 100 mL of RPMI-1640 medium containing PB (0.5 × MIC, 1 × MIC, and 2 × MIC) and TBF (1 × MIC) were prepared at a cell density of 2 × 10^4^~5 × 10^4^ CFU/mL. Following incubation in the shaking incubator at 35°C for 24 h, fungal cells were harvested by centrifugation at 2000 × g for 5 min and the upper suspensions were discarded. The wet weight of cell pellets was detected after washing twice with sterile distilled water. Each sample was added the lysing agent (25% potassium hydroxide ethanol solution) and mixed well. The sample was placed in a water bath at 80°C for 2 h, cooled to room temperature, and decanted into a separatory funnel. Then, sterols were extracted by the mixture of 2 mL sterile distilled water and 3 mL petroleum ether. The organic layer was moved to sterile tubes and evaporated to dryness in a water bath at 80°C. Finally, these dry products were dissolved in 5 mL methanol and obtained by filtrating through 0.22 *μ*m filters.

Corresponding prepared samples were separated and analyzed at 35°C by using a Venusil MP C18 analytical column (2.1 × 100 mm, 2.5 *μ*m). The mobile phase was methanol at a flow rate of 0.5 mL·min^−1^. Aliquots of 10 *μ*L were directly injected into HPLC for determination. The detection wavelength was set at 281 nm, calculating ergosterol content from the standard calibration curve using ergosterol as standard. The results were expressed as $\overset{¯}{\;x}\pm \text{SD}$. The equations for ergosterol content of wet vectors and ergosterol reduction rate were proposed as follows:

(1) $$\begin{array}{c} \text{Ergosterol content of wet vectors }\left(w\right)=\frac{\left(\text{peak area}+361.06\right)\times \text{dilution ratio}\times \text{sample size}}{6287\times \text{weight of wet vectors}}, \end{array}$$

(2) $$\begin{array}{c} \text{Ergosterol reduction rate}=\frac{\text{control group }\left(w\right)–\text{drug group }\left(w\right)}{\text{control group }\left(w\right)}\times 100\%. \end{array}$$

### 2.15. Estimation of Squalene Epoxidase (SE) and Sterol 14*α*-Demethylase (CYP51) Activities in T. rubrum Membrane

The effects of PB against SE and CYP51 activities were investigated by ELISA according to published protocols [35]. Fungal suspensions were diluted to the final inoculum of 2 × 10^4^~5 × 10^4^ CFU/mL by RPMI-1640 medium containing PB at 0.5 × MIC, 1 × MIC, and 2 × MIC. TBF is a positive drug for the detection of SE activity while MCZ is a positive drug for the detection of CYP51 activity. Cultures were incubated at 35°C under continuous shaking for 24 h. The fungal deposits were obtained using centrifugation after being washed three times with PBS (0.01 M, pH 7.2). The samples were suspended in extracting solution, sonicated on an ice bath, then frozen, and thawed twice more to extract SE and CYP51 enzymes. The supernatant was removed by centrifugation at 5000 × g for 5 min at 4°C. SE activity was determined strictly by a commercial kit assay kit (mLbio, Shanghai, China), and CYP51 activity was detected using a commercial kit assay kit (Biomart, Tianjin, China). The OD values at 450 nm were read using a microplate reader (Bio-Rad, CA, USA) within 15 min.

### 2.16. Statistical Analysis

IBM SPSS Statistics 21.0 software and GraphPad Prism version 8.0.2 were used to analyze data. Analysis of variance using one-way ANOVA was performed to test the difference between treated and untreated samples. Values were presented as mean ± standard deviation (*X* ± SD). Levels of statistical significance were set at ^∗^*p* < 0.05 and ^∗∗^*p* < 0.01.

## 3. Results

### 3.1. Antifungal Activity of Drugs against T. rubrum

MIC and MFC were used to determine the susceptibilities of *T. rubrum* to drugs and may be used in experiments to optimize the dosage regimen of antifungal drugs. The MIC of PB against *T. rubrum* was 20 *μ*g/mL, whereas MFC was 40 *μ*g/mL. The MIC and MFC of TBF on *T. rubrum* were 0.0625 *μ*g/mL and 0.125 *μ*g/mL, respectively. The MIC of AMB for *T. rubrum* was 0.5 *μ*g/mL, equivalent to MFC, and for *Candida parapsilosis* (ATCC 22019) was within the range specified in the CLSI reference documents (0.5~4 *μ*g/mL). Besides, both MIC value and MFC value of MCZ for *T. rubrum* (CMCC(F)T1d) were 0.25 *μ*g/mL.

### 3.2. Time-Kill Kinetics Analysis of PB against T. rubrum

In order to understand the rate of antidermatophyte activity, PB and TBF (positive control) were selected for time-killing kinetics assay. The time-killing curve of PB against *T. rubrum* (CMCC(F)T1d) is shown in Figure 2. At the concentrations of 0.5 × MIC and 1 × MIC, PB was fungistatic (less than 99.9% reduction or 3log_10_ in the CFU/mL versus the initial inoculum). However, a decrease in the population of *T. rubrum* reached 100% at 2 × MIC after 36 h treatment. Changes between fungistatic and fungicidal activity further revealed that PB had a concentration-dependent antifungal activity. In addition, TBF at 2 × MIC also exerted fungicidal activity up to 24 h.

### 3.3. Effect of PB on the Total Biomass of T. rubrum

The effects of PB on the total biomass of *T. rubrum* were determined by measuring the dry mycelia mass (Table 1). The results showed that TBF significantly inhibited mycelial growth of *T. rubrum*, compared with control group (*p* < 0.01). Additionally, the decreased rate of total biomass exposed to TBF at 1 × MIC was 54.12%. A dose-dependent inhibition of total biomass was noted in *T. rubrum* cells after PB treatment (*p* < 0.01). The total biomass was reduced by 64.17%, 77.65%, and 84.71% in the presence of PB at 0.5 × MIC, 1 × MIC, and 2 × MIC, respectively.

### 3.4. Effect of PB on the Apparent Morphology of T. rubrum

The apparent morphological structure of *T. rubrum* was observed by SEM. As illustrated in Figure 3(a), untreated *T. rubrum* showed the normal morphogenesis with smooth surfaces, plump hyphae, uniform cytoplasm, and good growth. The treatment of PB at 0.5 × MIC caused shrinkage of fungal filaments in *T. rubrum* (Figure 3(c)). When the concentration was increased to 1 × MIC, *T. rubrum* appeared distorted and severely collapsed due to the lack of cytoplasm (Figure 3(d)). Similar morphological changes were observed in the hyphae treated with 2 × MIC. Distorted hyphae seemed to be squashed and almost flattened (Figure 3(e)). TBF-treated cells also showed aberrant morphologies, which were consistent with the results of PB treatment (Figure 3(b)).

### 3.5. Effect of PB on the Internal Morphology of T. rubrum

The internal morphology of T. rubrum, with or without treatment with PB, was obtained by TEM. As shown in Figure 4(a), the untreated control T. rubrum exhibited the regular cell wall thoroughly surrounded by the unfolded cytoplasmic membrane with uniform shape in all parts. The cell matrix was homogenous with the structural integrity of organelles, including nuclei, mitochondria, and ribosome. In the presence of PB at 0.5 × MIC, morphological alternations in fungal compartments included abnormal distributions of polysaccharides in the cytoplasm and degradation of cytoplasmic content (Figure 4(c)). Folding and breaking down of the cytoplasmic membrane at numerous sites, as well as plasmolysis, were seen when *T. rubrum* was treated with PB at 1 × MIC (Figure 4(d)). Moreover, *T. rubrum* exposed to PB at 2 × MIC showed severe cell disruption and disarray, involving extensive organelle destruction and lysis, large cytoplasm vacuolation with vacuole fusion, and plasmalemma rupture (Figure 4(e)). Similar alternations were observed in TBF-treated cells (Figure 4(b)).

### 3.6. Effects of PB on the Cell Wall and Membrane of T. rubrum

Table 2 represented the results of broth microdilution method for PB against *T. rubrum*. In the sorbitol protection assay, the MIC values of PB remained unchanged compared to those without sorbitol. As for ergosterol binding assay, the MIC of PB was increased by 4-fold in the presence of exogenous ergosterol as compared to those without it. Similarly, the addition of exogenous ergosterol to the medium resulted in a 16-fold increase in the MIC of AMB (positive control). Fungal growth was observed in control.

### 3.7. Effect of PB on the Nucleotide Leakage

To examine the membrane damaging extent of PB against *T. rubrum*, the nucleotide leakage was tested. The results are shown in Figure 5. After 4 h and 8 h of medication therapy, AMB (positive control) induced obvious leakage of intracellular nucleotides as compared to the control group (*p* < 0.01). At different time intervals (4 h and 8 h), 0.5 × MIC, 1 × MIC, and 2 × MIC of PB increased the amount of nucleotide leakage with a concentration-dependent effect (*p* < 0.01).

### 3.8. Effect of PB on Ergosterol Content in T. rubrum Cell Membrane

The ergosterol content of *T. rubrum* cell membrane treated with PB at different concentrations was evaluated using an ultraperformance liquid chromatography (UPLC) method. The linear relationship between peak height (*y*) and ergosterol concentration (*x*) (4-40 *μ*g/mL) was good using the equation *y* = 6287*x* − 361.06, *r* = 0.9997. As seen in Table 3, compared with the control group, PB at different concentrations and TBF (positive control) induced an obvious decrease in ergosterol content of *T. rubrum*. Among them, the ergosterol content was decreased by 9.58%, 15.31%, and 76.24% in the presence of PB at 0.5 × MIC, 1 × MIC, and 2 × MIC, respectively. And the decreased rate of ergosterol content in 1 × MIC of TBF was 41.21%.

### 3.9. Effect of PB on Squalene Epoxidase (SE) Activity in T. rubrum Membrane

The effect of PB on SE activity was investigated by enzyme-linked immunosorbent assay (ELISA) using TBF as positive control. As illustrated in Figure 6, compared with the control group, TBF at 1 × MIC inhibited the SE activity in *T. rubrum* membrane (*p* < 0.01). Additionally, PB repressed the activity of SE enzyme in *T. rubrum* in a dose-dependent manner (*p* < 0.01).

### 3.10. Effect of PB on Sterol 14*α*-Demethylase Activity (CYP51) in T. rubrum Membrane

The effect of PB on CYP51 activity was investigated by ELISA using MCZ as positive control. The results are shown in Figure 7. Compared with the control group, MCZ at 1 × MIC had significant inhibition (*p* < 0.01) on CYP51 activity. Similarly, PB at 1 × MIC and 2 × MIC also caused an obvious reduction in the CYP51 activity (*p* < 0.01). The CYP51 activity in T. rubrum cells treated with PB at 0.5 × MIC was smaller than that of the control group but has no statistical significance (*p* > 0.05).

## 4. Discussion

*T. rubrum* is an anthropophilic specie that can get carbon, nitrogen, phosphorus, and sulfur from the host's nutritional macromolecules [4]. Since it overcomes the host defensive mechanisms, this is usually noticed among immunocompromised patients, particularly those undergoing bone marrow or solid organ transplantation. In addition, people with diabetes and hematological malignancies are at risk for fungal infection [36].

For decades, natural products and their phytochemicals have provided the basis for the vast majority of anti-infective therapies in clinical use, which are potential valuable source of new agents. *D. fragrans* is a traditional medicine fern used to treat dermatophytosis. Previous investigations have shown that the antifungal activity of this genus of plants is closely related to the amount of phloroglucinol [16, 37]. PB was isolated from phloroglucinol derivatives in aerial parts of *D. fragrans* [21] and possessed bioactivities due to interaction of its phenolic hydroxyl group and isobutyryl group with the hydrophobic tails of phospholipids [38]. In susceptibility tests, our data were in agreement with the previously reported results of antifungal activity of PB against dermatophyte strains in vitro (MIC range, 20 to 40 *μ*g/mL) [20]. Therefore, PB possesses great development potential and application prospects.

*T. rubrum* was submitted to the experimental approach for time-kill kinetics in order to characterize a dynamic connection between concentration and antidermatophyte activity over time. This assay has valuable therapeutic significance because it not only analyzes the duration of fungistatic action but also measures the fungicidal speed [33]. In this study, the time-kill curves exhibited that PB exerted 100% reduction in the population of *T. rubrum* at 2 × MIC after 36 h of incubation. TBF as a positive control showed a similar effect by 24 h. These results implied that PB could inhibit the growth of *T. rubrum*, which resembled those of Liu et al. [19], with regard to the decrease in the cell viability of *T. rubrum* after treatment with ethanol extracts of *D. fragrans* and TBF.

In the pathogenesis of dermatophytosis, filamentous hyphae were produced during the infection process, which exacerbated the damage and penetrated into the deeper keratinized tissues [8]. Thus, biomass does not reflect total living cells, but it shows the generation of fungal cell material [39]. Based on this perspective, the antifungal effect of PB against *T. rubrum* could be evidenced by our findings that PB treatment led to the reduction of mycelial biomass production. However, its possible antifungal mechanisms have not been elucidated and need to be further explored.

It has been reported that there is a significant correlation between morphological abnormalities and growth inhibition [40]. SEM images provide detailed view of cellular surfaces and damage, which can clearly show the difference between the treated and untreated *T. rubrum*. The hypha morphology of *T. rubrum* in the control group was normal and homogeneous with plump fungus and smooth surfaces. After being exposed to PB at 0.5 × MIC, the hyphae shrank and formed a rough surface, whereas those treated with PB at relatively higher concentrations (1 × MIC and 2 × MIC) were distorted, collapsed, and even flattened. According to the report [41], TBF could seriously destroy *T. rubrum* hyphae. This is consistent with our results of *T. rubrum* treated with TBF at 1 × MIC. SEM observation revealed that PB induced aberrant morphologies, which are essential for growth inhibition, cell viability, and virulence reduction.

TEM was regarded as an auxiliary technique to observe changes in the internal morphology of *T. rubrum* treated with PB [42]. The SEM results were further confirmed by TEM images. *T. rubrum* treated with PB showed abnormal distributions of polysaccharide particles, plasmolysis, degradation of organelles, and even excessive vacuolization accompanied by disintegration of cytoplasmic membrane. Our findings are in accordance with the previous investigations demonstrated below. The increase in hypha cell membrane permeability had been reported to give possible rise to plasmolysis [42]. As discussed by Zheng et al. [9], polysaccharide particles were derived from glycoproteins of damaged cell membranes. Therefore, cell membrane of *T. rubrum* was damaged by PB as a target.

The existing antifungal classes are mostly focused on the cell wall and membrane, in which the cell wall confers cell morphology against external osmotic shocks [43]. If drugs alter cell permeability, they might bring about an imbalance in osmotic pressure, subsequent autolysis and disorganization of intracellular organelles, depletion of cytoplasmic content, and finally cell death [44]. In general, the most major cellular modifications have been noted to include the breaking down of the cell wall and destruction and lysis of organelles, as well as damage to cell membrane permeability.

The sorbitol protection assay was performed to investigate whether PB acted on the fungal cell wall. This method used sorbitol as an osmotic protectant to stabilize fungal protoplasts [45]. Cell wall inhibitors share a special characteristic, where their antifungal activities are reversed in a medium plus sorbitol [33]. Consequently, MIC of cell wall inhibitors will shift to significantly greater values for the medium containing sorbitol. Nevertheless, the MIC values of PB were identical in the presence and absence of sorbitol. Other investigators also recorded the same results. For instance, as discussed by Danielli et al. [27], Schinus lentiscifolius Marchand essential oil could not change the MIC values of dermatophytes in the presence of sorbitol. These results proposed that the antifungal mechanism of PB was not associated with interfering with the cell wall of *T. rubrum*.

The cell membrane is a dynamic structure consisting of a lipid bilayer with enzymes and transport proteins embedded [46]. Since cell membrane of fungi in constituents and structures is different from mammalian, using it as a target is attractive for developing selective antifungal agents [47]. Currently, the majority of the available antifungals interfere with its functions either by binding with membrane ergosterol or through inhibition of various steps in ergosterol biosynthesis [48, 49].

AMB, a polyene antifungal drug, binds to the ergosterol in the fungal cell membrane and forms stable pores, producing membrane degradation and increased permeability. Small molecular substances and ions flow out of the cytoplasm, resulting in the death of fungi [50]. Ergosterol binding assay was performed to explore whether the medicine interfered with cell membrane. Exposure of fungi to cell membrane inhibitors leads to cell lysis in the absence of ergosterol, whereas fungi can grow in the presence of ergosterol. Thus, higher MIC values of drug used cell membrane as target would occur in the presence of exogenous ergosterol compared with the control group [51]. In this study, AMB showed an increase in its MIC of 16 times. The affinity of AMB with ergosterol in cell membrane was in agreement with the previous studies published [24]. In parallel, the MIC for PB increased 4-fold in the presence of exogenous ergosterol. The positive results further suggested that the mechanism of action of PB was related to the binding of ergosterol and subsequent instability of the fungal cell membrane.

In order to assess the degree of damage to cell membrane, *T. rubrum* was subjected to the method for nucleotide leakage. MOPS buffer is not capable of being degraded by cells and keeps *T. rubrum* in the stationary phase. Compounds with uracil, mainly nucleotides, release to the SDA medium from *T. rubrum* cells and exhibit the strongest absorption at 260 nm [52]. In this experiment, PB obviously amplified the nucleotide leakage of *T. rubrum* in a concentration-dependent manner after 4 or 8 h of incubation. Similar results were recorded in the studies concerning the effects of magnoflorine and AMB on the cellular material leakage of *T. rubrum* [53]. It suggested that the interaction of PB with cell membrane increased fluidity and permeability, causing cytoplasmic membrane degradation and loss in *T. rubrum*.

Cell membrane of fungi is enriched with diverse lipids, including glycerophospholipids, sphingophospholipids, and sterols [47]. Ergosterol is the primary sterol component of fungal cell membranes [39], involved in membrane permeability and fluidity modulation [52]. It also helps to maintain membrane structural integrity, cell viability, and material transportation [54]. A deficiency of ergosterol is indicative of interference in the ergosterol biosynthesis pathway. In this study, there were a dose-dependent decrease of ergosterol content in *T. rubrum* membrane after the treatment of PB. We speculated that disruption of ergosterol biosynthetic pathways might explain the mechanism of PB on fungal growth inhibition.

Ergosterol biosynthesis relates to a complex metabolic process. SE and CYP51 are among the key enzymes in the ergosterol biosynthesis pathway [53]. For most of fungi, SE is a flavin adenine dinucleotide (FAD) that catalyses the epoxidation of squalene to 2,3-oxidosqualene, thereby leading to a cascade of ergosterol biosynthetic pathways [55]. TBF is active when administrated either topically or orally. It is the most potent agent against dermatophytes and has a selective toxicity due to the greater sensitivity of fungal than mammalian squalene. In a classical known mechanism of action, TBF can specifically and selectively inhibit SE enzyme activity, resulting in depletion of ergosterol in fungal cell membrane (fungistatic effect) and the toxic accumulation of highly lipophilic squalene (fungicidal effect) [56]. In this study, a dose-dependent reduction in the activities of SE has been shown in *T. rubrum* treated with PB, preventing growth in a way similar to TBF.

Other major classes of antifungal agents take effects at later steps in the ergosterol biosynthesis pathway. For instance, MCZ acts by the inhibition of CYP51. This enzyme rests on activation of cytochrome P450, of which the active site is an iron protoporphyrin unit [57]. During its action, MCZ binds to the heme iron atom of cytochrome P450, preventing the oxidative removal of the lanosterol 14*α*-methyl group [58]. Therefore, the blockade of CYP51 causes accumulation of lanosterol and other 14a-methylated sterols in the cytoplasmic membrane of the fungi, inducing permeability change and malfunction of membrane proteins [59]. From this perspective, PB at MIC and 2MIC caused reduction in the CYP51 activity, which was comparable to the MCZ.

Methylphloroglucinol derivatives had been reported to reduce ergosterol content by inhibiting the activities of SE and CYP51 in *M. canis* [60]. This result corroborates with that presented above, which can justify ergosterol biosynthesis interference resulting from inhibition of sterol metabolism-related enzymes.

## 5. Conclusions

In summary, our study demonstrated that PB derived from aerial parts of *D. fragrans* could inhibit the growth of *T. rubrum* and induce the morphological alternations. The active target of PB was not the cell wall, but cytoplasmic membrane. PB primarily exerted antifungal activities not only by binding to ergosterol in cell membrane but also by lowering the ergosterol biosynthesis. Operation of these two modes of action altogether by PB could be very beneficial to combating infections caused by *T. rubrum*. However, the toxicity of PB plays a significant role in the clinical application. In order to develop a potential treatment of dermatophytosis for PB, more attention has been focused on the therapeutic benefits and safety on animal models.

## Figures and Tables

**Figure 1:** Structure and key HMBC correlations (H→C) of isoflavaspidic acid PB extracted from aerial parts of *Dryopteris fragrans* (L.) Schott.

**Figure 2:** Time-kill curve for *T. rubrum* (CMCC(F)T1d) after exposure to isoflavaspidic acid PB (0.5 × MIC: 10 *μ*g/mL; 1 × MIC: 20 *μ*g/mL; and 2 × MIC: 40 *μ*g/mL) and terbinafine (2 × MIC: 0.125 *μ*g/mL) (TBF: terbinafine; PB: isoflavaspidic acid PB). The log_10_CFU/mL is plotted versus time. Data were expressed as mean values ± standard deviation from three independent experiments.

**Figure 3:** Scanning electron micrographs of *T. rubrum* (CMCC(F)T1d) exposed to isoflavaspidic acid PB and terbinafine. (a) Control group (drug free); (b) terbinafine (1 × MIC: 0.0625 *μ*g/mL); (c) isoflavaspidic acid PB (0.5 × MIC: 10 *μ*g/mL); (d) isoflavaspidic acid PB (1 × MIC: 20 *μ*g/mL); (e) isoflavaspidic acid PB (2 × MIC: 40 *μ*g/mL).

**Figure 4:** Transmission electron micrographs of *T. rubrum* (CMCC(F)T1d) exposed to isoflavaspidic acid PB and terbinafine. (a) Cross-section of *T. rubrum* hyphae in the control group (drug free) indicated bilateral cell wall with intact edges, the outer cell wall (OCW) and the inner cell wall (ICW), uniform cytoplasm, nucleus (N), and clearly visible mitochondria (M); (b) cross-section of hyphae exposed to terbinafine (1 × MIC: 0.0625 *μ*g/mL) showed disorganization and degradation of cytoplasmic content (1); (c) cross-section of hyphae exposed to isoflavaspidic acid PB (0.5 × MIC: 10 *μ*g/mL) exhibited abnormal distributions of polysaccharides in the cytoplasm (2) and demolition of the endomembrane system (3); (d) cross-section of hyphae exposed to isoflavaspidic acid PB (1 × MIC: 20 *μ*g/mL) displayed cell membrane damage and cytoplasm shrinkage away from the cell wall (4). The medullary bodies and protein coagulators (5) were conspicuous in the cytoplasm (manifestations of apoptosis); (e) cross-section of hyphae exposed to isoflavaspidic acid PB (2 × MIC: 40 *μ*g/mL) had intact cell wall, uneven cytoplasmic density, blurred organelles, and excessive vacuolization (6). MIC: minimum inhibitory concentration. Bar represents 500 nm. Images were shown as 12000x magnification.

**Figure 5:** Rate of nucleotide leakage from *T. rubrum* (CMCC(F)T1d) treated with isoflavaspidic acid PB (0.5 × MIC: 10 *μ*g/mL; 1 × MIC: 20 *μ*g/mL; 2 × MIC: 40 *μ*g/mL) and amphotericin B (1 × MIC: 0.5 *μ*g/mL). AMB: amphotericin B; PB: isoflavaspidic acid PB. Lysing agent induced 100% of nucleotide release. Rate of nucleotide leakage was computed by comparing the test values with the lysing agent values. ^∗^*p* < 0.05 and ^∗∗^*p* < 0.01 versus the control group.

**Figure 6:** Effect of isoflavaspidic acid PB (0.5 × MIC: 10 *μ*g/mL; 1 × MIC: 20 *μ*g/mL; 2 × MIC: 40 *μ*g/mL) and terbinafine (1 × MIC: 0.0625 *μ*g/mL) on the activity of squalene epoxidase in *T. rubrum* membrane. TBF: terbinafine; PB: isoflavaspidic acid PB. Data were expressed as mean ± SD from three independent experiments. ^∗^*p* < 0.05 and ^∗∗^*p* < 0.01 versus the control group.

**Figure 7:** Effect of isoflavaspidic acid PB (0.5 × MIC: 10 *μ*g/mL; 1 × MIC: 20 *μ*g/mL; 2 × MIC: 40 *μ*g/mL) and miconazole (0.25 *μ*g/mL) on the activity of sterol 14*α*-demethylase in *T. rubrum* membrane. MCZ: miconazole; PB: isoflavaspidic acid PB. Data were expressed as mean ± SD from three independent experiments. ^∗^*p* < 0.05 and ^∗∗^*p* < 0.01 versus the control group.

**Table 1:** Effect of isoflavaspidic acid PB and terbinafine on total biomass of *T. rubrum*.

Group	Dosage (*μ*g/mL)	Total biomass (g)	Decrease rate of total biomass (%)
Control	—	0.085 ± 0.005	—
TBF 1 × MIC	0.0625	0.039 ± 0.006^∗∗^	54.12
PB 0.5 × MIC	10	0.030 ± 0.005^∗∗^	64.71
PB 1 × MIC	20	0.019 ± 0.002^∗∗^	77.65
PB 2 × MIC	40	0.013 ± 0.002^∗∗^	84.71

MIC: minimum inhibitory concentration; TBF: terbinafine; PB: isoflavaspidic acid PB. ^∗^*p* < 0.05 and ^∗∗^*p* < 0.01 versus the control group.

**Table 2:** MIC values (*μ*g/mL) of drugs in the absence and presence of sorbitol (0.8 M) and ergosterol (400 *μ*g/mL) against *T. rubrum* (CMCC(F)T1d).

Drug	Sorbitol			Ergosterol	
	Absence	Presence	Control	Absence	Presence
Isoflavaspidic acid PB	20	20	+	20	80
Amphotericin B^a^	—	—	+	0.5	8

^a^Positive control. (—): amphotericin B was not tested in the sorbitol assay. (+): fungal growth in the presence of sorbitol (0.8 M) and absence of drugs.

**Table 3:** Effect of isoflavaspidic acid PB and terbinafine on ergosterol content of *T. rubrum*.

Group	Dosage (*μ*g/mL)	Ergosterol content (*μ*g/g)	Decrease rate of ergosterol content (%)
Control	—	370.20 ± 1.46	—
TBF 1 × MIC	0.0625	217.63 ± 3.18^∗∗^	41.21
PB 0.5 × MIC	10	334.74 ± 7.67^∗∗^	9.58
PB 1 × MIC	20	313.51 ± 7.55^∗∗^	15.31
PB 2 × MIC	40	87.95 ± 11.16^∗∗^	76.24

MIC: minimum inhibitory concentration; TBF: terbinafine; PB: isoflavaspidic acid PB. ^∗^*p* < 0.05 and ^∗∗^*p* < 0.01 versus the control group.

## Data Availability

The data used to support the findings of this study are included within the article and are available from the corresponding author upon request. The spectroscopic data of compound is available at doi:10.7501/j.issn.0253-2670.2017.03.003.
